# Effect of Joint Use of External Minifixator and Titanium Lockplate on Total Active Motion Range and Hand Function Recovery in Comminuted Metacarpal and Phalanx Fracture Patients

**DOI:** 10.1155/2022/3566364

**Published:** 2022-01-25

**Authors:** Yao Li, Hongwei Zhang

**Affiliations:** Department of Orthopeadic Surgery, The First Affiliated Hospital of Jiamusi University, Jiamusi 154003, Heilongjiang, China

## Abstract

**Objective:**

To explore the effect of joint use of external minifixator and titanium lockplate on total active motion (TAM) range and hand function recovery in comminuted metacarpal and phalanx fracture patients.

**Methods:**

The medical data of 70 patients with comminuted metacarpal and phalanx fracture treated in our hospital from June 2017 to June 2020 were screened for the retrospective study, and the patients were divided into the control group (Kirschner wire internal fixation) and the study group (an external minifixator with titanium lockplate) according to the treatment modalities, with 35 cases each. After treatment, the clinical efficacy of patients was compared between the two groups.

**Results:**

No between-group differences in patients' general data were observed (*P* > 0.05); the time for hospital stay and fracture healing was obviously shorter in the study group than that in the control group (*P* < 0.05); after treatment, the study group obtained significantly higher TAM range good rate (*P* < 0.05), significantly higher Carroll hand function test pass rate (*P* < 0.05), and obviously better grip strength of both hands and score on digital opposition of thumb than those in the control group (*P* < 0.05); and after surgery, the study group had significantly lower incidence rates of complications such as infection, local inflammation, displacement of bone, and adhesion of tendon that those in the control group (*P* < 0.05).

**Conclusion:**

Joint use of an external minifixator and titanium lockplate can effectively promote the TAM range and accelerate hand function recovery for comminuted metacarpal and phalanx fracture patients and is conducive to reducing the incidence of postoperative complications, which is safe and has significant efficacy.

## 1. Introduction

The hand is the most flexible and applied organ in the human body, so the fractures of palms and phalanges are also relatively common in daily life, with an incidence of about 10% of all fractures [1–4]. According to clinical statistics, most of the comminuted metacarpal and phalanx fractures are caused by trauma and require emergency treatment, so selecting a correct and effective treatment modality in the acute treatment period is extremely important for the recovery of hand function of patients. Hands are characterized by multiple joints as well as fine and complex muscles and tendons, and the injuries are combined with unstable fracture blocks, which, combined with mixed injuries of nerves, tendons, and blood vessels, increases the difficulty in the treatment of comminuted metacarpal and phalanx fractures [5–8]. However, the traditional treatment of debridement and internal fixation with Kirschner wires has the risks of slow fracture healing, long fixation time, late functional exercise, and poor fracture stability associated with wound skin necrosis, bone exteriorization, tendon adhesion, and soft tissue contracture, leading to poor postoperative hand functional recovery and suboptimal clinical outcomes. In recent years, as the application efficacy of an external minifixator and titanium lockplate has been confirmed at home and abroad, its use in clinical treatment has become more widespread. At present, the related studies in this field are mostly around clinical cases for summary analysis, and there are few comparative studies. A total of 70 patients with comminuted metacarpal and phalanx fracture treated in our hospital from June 2017 to June 2020 were screened for the retrospective study, among which 35 cases were treated by using an external minifixator with titanium lockplate and showed higher satisfaction with clinical efficacy at postoperative follow-up. The study results were summarized as follows.

## 2. Study Plan

### 2.1. Cases Screening and Grouping

The medical data of 70 cases with comminuted metacarpal and phalanx fracture treated in our hospital from June 2017 to June 2020 were screened for the retrospective study, and the patients were divided into the control group and study group according to the treatment modalities, with 35 cases each. The study plan was strictly reviewed and approved by the hospital ethics committee.

### 2.2. Inclusion Criteria

① All patients were diagnosed with comminuted metacarpal and phalanx fracture via imaging examinations including X-ray, CT, or MRI, ② the patients had complete clinical data, ③ the patients and their family members were informed of and agreed to join the study, ④ the patients had comminuted fracture of single palm, and ⑤ before surgery, the patients had normal hand motion and did not have a history of long-term numbness or pain.

### 2.3. Exclusion Criteria for Patients

① Pathological fracture (which is mainly caused by the primary disease, and treatment options should be specifically analyzed according to the primary disease, not with respect to fracture symptoms alone), ② complicated with other severe organic diseases or malignancies, ③ cognitive disorder, seeing-hearing disorder, or other limb activity disorder, ④ history of comminuted metacarpal and phalanx fracture, ⑤ suffering from rheumatic immune disease, ⑥ long-term use of hormones, and ⑦ poor treatment compliance.

### 2.4. Methods

Patients in the control group received the Kirschner wire internal fixation treatment, and those in the study group were treated with an external minifixator with a titanium lockplate.

For patients with closed fracture, brachial plexus block was performed; an arc incision was made at the dorsal metacarpophalangeal joint or interphalangeal joint, and an s-shaped incision was made at the distal interphalangeal joint; the extensor tendon was cut open longitudinally, and the articular capsule was cut open horizontally to fully expose the fracture end; according to the fracture status of patients during surgery, the sequence of reduction, then internal fixation with a titanium lockplate, and installation of an external minifixator (manufactured by Orthofix) was determined; for patients in the control group, only internal fixation with the Kirschner wire (model: 1.0*∗*150; manufactured by Changzhou Ai Men Medical Instrument Co., Ltd.) was performed [8–11]. For patients with an open fracture, after observing the open wound, the incision could be extended appropriately as needed to fully expose the fracture end; the extensor tendon should be cut open longitudinally if there was no injury; the sequence and methods for installation of an external minifixator and reduction and then internal fixation with a titanium lockplate were the same as those for closed fracture; and in case of injured collateral ligament or articular capsule, repair should be performed during operation.

Installation of the external minifixator is as follows: the external fixator was installed across the joint, the 1st fixing pin was inserted proximal to the fracture, and the 2nd fixing pin was inserted along a parallel hole on the 1st pin clamp, and a C-arm was used to confirm that the tip of the fixing pin was exactly through the contralateral cortical bone. The 3rd and 4th fixing pins were inserted sequentially at the distal fracture along a parallel hole on the 2nd pin clamp, and the clamp was kept at a distance of 5–10 mm from the skin. It should be noted that the ball-and-socket joint in the center of the external fixator was at the same level as the joint space of the damaged joint. The joint space was expanded 1.5–2 mm to confirm the fracture reduction status and the installation position of the external fixator by C-arm, and then, all bolts were fixed. For intra-articular fracture of the thumb, the fixing pin was inserted on the side central line at the radial thumb. For intra-articular fracture of the index finger, middle finger, and ring finger, the fixing pin should be inserted at a 45° angle from the dorsoradial branch to the horizontal plane; also, it could be inserted at a 45° angle from the dorsoulnar branch to the horizontal plane for intra-articular fracture of the middle finger and ring finger [12–14]. For intra-articular comminuted fracture of the little finger, the fixing pin was inserted on the side central line of the ulnar branch of the little finger.

Specific operation for reduction, then internal fixation with titanium lockplate is as follows: reconstruction of the fracture end was performed under direct viewing; a mini-titanium plate was placed lateral or dorsal to metacarpophalangeal bones and fixed by drilling holes and screwing into bolts. For metacarpal and phalanx diaphyseal transverse and oblique fracture, a straight titanium plate was selected for pressurized fixing; for fracture of metacarpal and phalanx basilar part and head, bolts and Kirschner wire were chosen for the fixation of free fragments and fractured fragments; and for metacarpal and phalanx basilar part and head intra-articular fracture, a T-shaped or L-shaped titanium plate was selected for the fixation.

### 2.5. Observation Indexes

General data: patients' data including age, BMI, fractured site, fracture type, cause of fracture, and gender were recorded for statistics; and after treatment, follow-up was conducted to patients, and their hospital stay and fracture healing time were recorded for statistics. The postoperative complications in patients of the two groups were recorded for statistics.

Patients' finger function after treatment was assessed by using the Total Active Flexion (TAF) scale [15] with the active flexion from the metacarpophalangeal joint to the interphalangeal joint of digit 2–5 being the reference, >220° meant excellent, 180–220° meant good, and <180° meant poor, and the good rate of each group = (number of excellent cases + number of good cases)/total number × 100%. The Carroll hand function test [16] was one of the more reliable methods to comprehensively assess patients' hand function, which contained 33 items. Each item was rated on a scale of 0–3 points, and the maximum score for the dominant hand and nondominant hand was, respectively, 99 points and 96 points. A score of 90 points and above indicated normal function, 76–89 points indicated imperfect hand function, 76 points and above indicated passing the Carroll hand function test, and less than 75 points indicated severe hand dysfunction.

Grip strength of both hands. Patients' grip strength of both hands was measured with the hand dynamometer and pinch-grip dynamometer in kg.

Score on digital opposition of thumb [17]. The patients' finger function was assessed according to whether the thumb of their affected hand could touch the index finger, middle finger, ring finger, and little finger of the same hand. It was rated by the farthest part the thumb could get, with 1–5 points, respectively, referring to touching the tip of the index finger, tip of the middle finger, tip of the ring finger, tip of the little finger, and the transverse palmar creases on the proximal-distal aspect of the little finger, and 0 point referring to the failure to touch the index finger.

### 2.6. Statistical Processing

In this study, the between-group differences in data were calculated by using SPSS22.0, the picture drawing software was GraphPad Prism 7 (GraphPad Software, San Diego, USA), the items included were enumeration data and measurement data, which were expressed by [*n*(%)] and ($\bar{x}\pm s$) and examined by *X*^2^ test and *t*-test, respectively, and differences were considered statistically significant at *P* < 0.05.

## 3. Results

### 3.1. General Data

No statistical differences in patients' general data including age, BMI, fractured part, fracture type, cause of fracture, and gender were observed (*P* > 0.05). See Table 1.

### 3.2. Total Active Motion (TAM) Range

After treatment, the TAM range good rate was significantly higher in the study group than in the control group (*P* < 0.05), presenting statistically significant difference. See Table 2.

### 3.3. Clinical Treatment

The study group had obviously shorter hospital stay and fracture healing time than the control group (*P* < 0.05). See Table 3.

### 3.4. Carroll Hand Function Assessment

After treatment, the pass rate of the Carroll hand function test was significantly higher in the study group than that in the control group (*P* < 0.05). See Figure 1.

### 3.5. Grip Strength of Both Hands and Digital Opposition of the Thumb

According to the statistics in Table 4, patients' grip strength of both hands and the score on digital opposition of the thumb after treatment were significantly better in the study group than those in the control group (*P* < 0.05).

### 3.6. Postoperative Complications

The incidence rates of postoperative complications including infection, local inflammation, displacement of bone, and adhesion of tendon were significantly lower in the study group than those in the control group (*P* < 0.05). See Table 5.

## 4. Discussion

Metacarpophalangeal joints are highly specific to other parts, and metacarpal and phalanx are composed of short tubular bones with multiple joints and complex surrounding structure of the bone and are highly functionally demanding and topographically influencing, thus requiring timely implementation of functional exercises to promote early rehabilitation [18, 19]. Hence, comminuted metacarpal and phalanx fractures are more difficult to treat than fractures of long tubular bones of the extremities. The basic configuration of an external minifixator is unilateral, easy to operate, and less traumatic to the body, which has the following advantages: it does not affect the fracture end but enables transarticular fixation; it has little effect on soft or tendon tissues; it can adjust reduction by traction, distract to restore the joint space, and reduce the incidence of traumatic arthritis; it may promote fracture healing by adjusting compression; and it can assist the fixation of open fractures. Therefore, an external minifixator can maintain alignment between the joint and fracture site by adjusting the direction of the universal joint so as to fully adjust the fracture site during the process of reduction and healing, and if the displacement of bone is found, it can be promptly adjusted to achieve fracture reduction. The connection bar of the external minifixator has a longitudinal extrusion effect, which can maintain tight junction of the fracture site, produce stress stimulation, and promote bone cell growth, making its fixation to the fracture end more stable and reliable. Moreover, it is of elastic fixation, and the axial stress change of the fracture site can effectively stimulate the growth of bone callus and promote fracture healing, so the external minifixator is flexibly operative for external fixation and stable and solid for internal fixation. In addition to its convenience in operation, an external minifixator can protect soft tissue, reduce vascular damage, guarantee the blood circulation of covered skin, and reduce the probability of osteomyelitis induced by bone nonunion and infection in severe cases of open soft tissue injury [13, 17, 20, 21]. An external minifixator is able to promote fracture healing, so patients can perform rehabilitation exercises and joint motion as early as possible to avoid the occurrence of joint deformity, stiffness, and other conditions. The titanium lockplate does not go through joints for fixation and is easy to operate and secure, and by jointly using the external minifixator, the healing rate can be greatly accelerated, so that patients can perform active and passive functional exercises after surgery, which is beneficial for reducing edema and bone atrophy that occur after hand trauma and of great significance particularly for performing early rehabilitation exercise of adjacent metacarpophalangeal and finger joints, promoting the early healing and functional recovery of the fracture. The lockplate compensates for the disadvantages such as easy slippage and loosening, unfavorable anatomical reduction, easy separation of fracture ends, and limiting early functional exercises of internal fixation with Kirschner wires. In addition, it occupies less space and has less influence on the activity of surrounding tissues, especially tendons. In summary, titanium lockplate is significantly superior to other internal fixation methods in terms of surface stiffness, stability, and pressure. However, for distal fractures with not enough space for the application of fixation materials which can cause the decrease in stability, the external minifixator can be jointly applied.

The study concluded that the hospital stay and fracture healing time were obviously shorter in the study group than the control group (*P* < 0.05), which was consistent with the study by Katayama et al. [22], further demonstrating that performing treatment to patients with comminuted metacarpal and phalanx fracture by using an external minifixator and titanium lockplate could effectively promote fracture healing, laying a good foundation for subsequent rehabilitation and treatment, and shortening patients' hospital stay. Moreover, after treatment, the TAM range good rate, Carroll hand function test pass rate, grip strength of both hands, and the score on digital opposition of thumb were significantly higher in the study group than the control group (*P* all < 0.05), which proved that the external minifixator and titanium lockplate had active effect on recovery of hand function and TAM range for patients with comminuted metacarpal and phalanx fracture. Finally, the incidence rates of postoperative complications including infection, local inflammation, displacement of bone, and adhesion of tendon were significantly lower in the study group than in the control group (*P* < 0.05), indicating that joint application of an external minifixator and titanium lockplate had a good fixation effect and stability and higher safety, so patients could perform hand function exercises after surgery as early as possible and suffer from fewer complications.

In conclusion, joint use of an external minifixator and titanium lockplate can effectively promote the TAM range and accelerate hand function recovery of patients with comminuted metacarpal and phalanx fracture and is conducive to reducing the occurrence of postoperative complications, with significant efficacy and higher safety. However, the sample size of the study was smaller, so the conclusion should be further proved by subsequent studies with a larger sample size; in addition, the study had a short follow-up time for patients, whereas metacarpophalangeal fractures required a longer recovery time, so extended follow-up time is still needed in subsequent related studies to comparatively analyze the long-term outcomes of an external minifixator combined with titanium lockplate for comminuted metacarpophalangeal fractures.

## Figures and Tables

**Figure 1:** Carroll hand function test results of the two groups (%). The horizontal axis indicated the groups, and the vertical axis indicate the percentage. In the control group, 15 cases passed the Carroll hand function test. In the study group, 26 cases passed the Carroll hand function test. ^*∗*^indicates a significant difference in the Carroll hand function test pass rate between the two groups (*X*^2^ = 7.124, *P*=0.008).

**Table 1:** Between-group comparison of patients' general data (*n* = 35).

Observation indicator	Control group	Study group	*X* ^2^/*t*	*P* value
Age (years)	36.57 ± 5.10	37.00 ± 6.61	−0.304	0.762
BMI (kg/m^2^)	22.95 ± 3.00	24.49 ± 4.14	−1.773	0.081
Fractured part			0.058	0.810
Metacarpal bone	16 (45.71%)	15 (42.86%)		
Digital bone	19 (54.29%)	20 (57.14%)		
Fracture type			0.068	0.794
Open fracture	11 (31.43%)	10 (28.57%)		
Closed fracture	24 (68.57%)	25 (71.43%)		
Cause of fracture			0.273	0.872
Injury by heavy crashing object	9 (25.71%)	8 (22.86%)		
Injury by machine	16 (45.72%)	15 (42.85%)		
Injury by exercise	10 (28.57%)	12 (34.29%)		
Gender			0.280	0.597
Male	24 (68.57%)	26 (74.29%)		
Female	11 (31.43%)	9 (25.71%)		

**Table 2:** Between-group comparison of patients' TAM range [*n*(%)].

Group	Poor	Good	Excellent	Good rate
Study (*n* = 35)	1 (2.86)	17 (48.57)	17 (48.57)	34 (97.14)
Control (*n* = 35)	9 (25.71)	14 (40)	12 (34.29)	26 (74.29)
*X* ^2^				7.552
*P* value				0.023

**Table 3:** Patients' hospital stay and fracture healing time ($\bar{x}\pm s$).

Group	*n*	Hospital stay (d)	Fracture healing time (months)
Control	35	14.91 ± 3.10	5.99 ± 1.58
Study	35	7.96 ± 2.83	2.85 ± 0.56
*t*		9.807	11.048
*P* value		<0.001	<0.001

**Table 4:** Grip strength of both hands and digital opposition of the thumb ($\bar{x}\pm s$).

Group	*n*	Grip strength of both hands (kg)	Score on digital opposition of the thumb
Control	35	10.41 ± 3.41	3.95 ± 0.61
Study	35	13.69 ± 3.51	4.86 ± 0.53
*t*		−3.961	−6.645
*P* value		<0.001	<0.001

**Table 5:** Between-group comparison of postoperative complication incidence [*n*(%)].

Group	Infection	Local inflammation	Displacement of bone	Adhesion of tendon	Total incidence rate
Study	0 (0)	2 (5.71)	0 (0)	0 (0)	2 (5.71)
Control	1 (2.86)	3 (8.57)	2 (5.71)	3 (8.57)	9 (25.71)
*X* ^2^					5.285
*P* value					0.022

## Data Availability

The data to support the findings of this study are available on reasonable request from the corresponding author.
